The article "Association of Serum Apolipoprotein A5 Concentration with Nonalcoholic Fatty Liver Disease in Ningbo, China" was published in 2022. Journal: Contrast Media Mol Imaging.

# Association of Serum Apolipoprotein A5 Concentration with Nonalcoholic Fatty Liver Disease in Ningbo, China

**DOI:** 10.1155/2022/7015528

**Published:** 2022-07-08

**Authors:** Xiao Liu, Ping Xu, Xueping Tao, Wenli Li, Qiongyi Hong, Qunfen Cao

**Affiliations:** ^1^Department of Gastroenterology, The Ningbo Seventh Hospital, Ningbo 315200, China; ^2^Department of Ultrasound, Ningbo Yinzhou No. 2 Hospital, Ningbo 315199, China

## Abstract

Nonalcoholic fatty liver disease (NAFLD) is a common chronic disease characterized by the excessive accumulation of hepatocyte fat and steatosis in the absence of alcohol or any other clear contributing factors to liver injury. NAFLD has been confirmed to be closely associated with obesity, insulin resistance, and dyslipidemia. Genetic polymorphism studies have shown the relations between the apolipoprotein A5 gene (APOA5) and NAFLD. However, the association between the serum ApoA5 level and NAFLD remains unclear. Between September 2018 and August 2019, adults who attended the hospital-based health checkup center were enrolled in this study. Anthropometric examination, laboratory investigations on fasting blood, and abdominal ultrasonography were performed. The serum ApoA5 level was determined by enzyme-linked immunosorbent assay. A total of 517 eligible participants (317 females and 200 males) were involved in this study, with a mean age of 54.7 ± 16.7 years. The mean ApoA5 concentration was 28.8 ± 4.7 *μ*g/ml, among which the males had higher concentration levels than females (29.3 ± 4.5 vs. 28.5 ± 4.7 *μ*g/mL, *P*=0.04). Serum ApoA5 level was not significantly correlated with NAFLD or metabolic profiles. However, the prevalence rate of hypertriglyceridemia (triglyceride ≥ 1.7 mmol/L) showed a significant inverted “U”-shaped trend in individuals with the serum ApoA5 level of quartile one to quartile four after adjusting the confounding factors. Moreover, individuals with higher serum ApoA5 levels were also more likely to suffer from hyperglycemia. The ApoA5 levels and the prevalence of hypertriglyceridemia are in an inverted “U-shaped” correlation, but there is no significant difference between ApoA5 levels, NAFLD, and metabolic syndrome.

## 1. Introduction

Nonalcoholic fatty liver disease (NAFLD) is a common chronic disorder characterized by the excessive accumulation of hepatocellular fat and steatosis, which is in the absence of alcohol or any other definite liver damage factors [1–3]. NAFLD has been confirmed to be closely related with obesity, insulin resistance, and dyslipidemia. Meanwhile, just because of this, it is considered to be liver manifestation of the metabolic syndrome and is often accompanied by an increased risk of type 2 diabetes and cardiovascular diseases [4, 5]. With a worldwide prevalence of nearly 25%, NAFLD seriously threatens the global economy and health care system [2, 6–10].

The ApoA5 gene is located in the apolipoprotein gene (ApoA1/C3/A4/A5) cluster on human chromosome 11q23, a locus which is well known for its role in the lipid metabolism [11, 12]. Apolipoprotein A5 (ApoA5), a novel apolipoprotein and a key regulator of the serum triglyceride derived from the ApoA5 gene, has been confirmed to be specially expressed in the hepatocellular cells, and it is secreted into the serum at a low concentration [11, 13–15]. Since its discovery in 2001, numerous studies have shown that ApoA5 plays a crucial role in triglyceride (TG) metabolism and has attracted increasing attention owing to its multifunction in several target organs [11, 15–19]. For instance, through comparative sequencing, ApoA5 was shown to affect the triglycerides in both humans and mice. Importantly, the serum TG levels in ApoA5-deficient mice showed a 4-fold increase, whereas its levels were remarkably decreased in ApoA5 overexpressed mice [11]. Studies have also reported that the expression of the ApoA5 mRNA in NAFLD patients was significantly increased in the liver [20]. Moreover, a genetic polymorphism study in the Chinese population also demonstrated a correlation between the metabolic control and ApoA5 gene in patients with NAFLD [21], but whether the serum ApoA5 level is associated with metabolic syndrome and NAFLD remains unknown.

The serum ApoA5 level of the patients enrolled in this study was detected to investigate whether there is an association between the serum ApoA5 level, metabolic syndrome, and NAFLD in the general population of China.

## 2. Materials and Methods

### 2.1. Study Design and Human Subject Collection

A total of 517 human subjects (200 males and 317 females)recruited in this study were obtained from the health check center of the Ningbo Seventh Hospital, Ningbo, China, from September 2018 to August 2019. All the subjects who were initially enrolled had complete health records on anthropometric examination, laboratory testing, and abdominal ultrasonography. NAFLD diagnosis was performed under the conditions of standard clinical evaluation following the Asia-Pacific Working Party criteria. The exclusion criteria were as follows: (1) alcohol consumption >140 g/week for males and >70 g/week for females; (2) a history of viral hepatitis, drug-induced hepatitis, autoimmune hepatitis, and/or other forms of chronic liver disease or if currently on hepatotoxic medication; (3) body mass index (BMI) <18.5 kg/m^2^. Written consent was submitted by all individual participants enrolled in this study.

### 2.2. Biochemical Analyses and Serum ApoA5 Detection

After a night of fasting for at least 8 hours, a comprehensive test was conducted in the morning. Then, the body weight, height, waist circumference, and blood pressure of the enrolled patients were measured according to the standard protocol, and the anthropometric measurements data were collected.

Next, the fasting serum glucose (FPG), total cholesterol, TG, HDL-cholesterol (HDL-C), LDL-cholesterol (LDL-C), urine acid, serum alanine aminotransferase (ALT), aspartate aminotransferase (AST), and serum ApoA5 level were further tested. Additionally, the serum ApoA5 level from each sample was tested using the human ApoA5 ELISA kit (Jianglai Biotech, Shanghai, China) under the guidance of the manufacturer's instruction.

### 2.3. Ultrasonography and NAFLD Diagnosis

The hepatic ultrasonic examination was conducted by two trained ultrasonographists using a Toshiba Nemio 20 sonography machine (Toshiba, Tokyo, Japan) with a 3.5-MHz probe. NAFLD was diagnosed based on the ultrasound image with evidence of hepatic steatosis after excluding the significant alcohol consumption, hepatitis B/C, medication use, hereditary disorders, or any other definite liver damage factors.

### 2.4. Metabolic Syndrome Definition

The metabolic syndrome was defined according to the national cholesterol education program (NCEP) and the adult treatment panel III (ATP III) criteria [22, 23]. If at least three or more of the following five criteria were met, the metabolic syndrome was considered: (1) central obesity: waist circumference ≥90 cm in men and ≥80 cm in women; (2) hypertriglyceridemia: fasting TG ≥1.7 mmol/L; (3) low HDL-C: fasting HDL-C <1.03 mmol/L for men and <1.29 mmol/L for women; (4) hypertension: BP ≥130/85 mmHg and/or on antihypertensive drugs; and (5) hyperglycemia: FPG ≥5.6 mmol/L or previously diagnosed type 2 diabetes.

### 2.5. Statistical Analyses

Based on a cross-sectional study, the association between the serum ApoA5 level, metabolic syndrome, and NAFLD were estimated. The SPSS software package (version 18.0, IBM, USA) was employed for statistical analysis. The continuous variables were presented as the mean ± standard deviation (SD) or median (interquartile range) as appropriate, whereas the category variables were presented as number (%). Student's *t*-test and *χ*^2^-test (for categorical variables) were used for group comparisons flexibly according to the conditions. To determine the correlation between the ApoA5 level and metabolic profiles (as continuous value), Pearson correlation analysis was conducted. Furthermore, the associations between the quartiles of the ApoA5 levels and the metabolic control evaluation were analyzed on the basis of the general linear model or the logistic regression analysis method. *P* < 0.05 (2-tailed test) was considered statistically significant.

## 3. Results

### 3.1. Characteristics of Subjects

A total of 517 eligible subjects (200 males and 317 females, mean age: 54.7 ± 16.7 years) with a mean serum ApoA5 level of 28.8 ± 4.7 *μ*g/mL were enrolled. Among them, 139 individuals (26.9%) were considered to have metabolic syndrome and 136 individuals (26.3%) were diagnosed with NAFLD.

### 3.2. The Association between ApoA5 Level and Gender and Metabolic Characteristics

In this study, the associations between the ApoA5 level and the gender of participants were explored. Our data indicated that the serum ApoA5 level was significantly higher in men than in women (29.3 ± 4.5 vs. 28.5 ± 4.7 *μ*g/mL, *P*=0.04). However, no significant difference was observed in the serum ApoA5 level in patients with or without NAFLD or metabolic syndrome. Subsequently, we further analyzed the relationship between the different components of the metabolic syndrome and the levels of ApoA5. As shown in Table 1, the individuals with hyperglycemia tend to have a higher ApoA5 level, but the difference was not statistically significant (29.4 ± 4.8 vs. 28.6 ± 4.6 *μ*g/mL, *P*=0.075). Similarly, there were no significant differences observed in the serum ApoA5 level between those with or without hypertension, hypertriglyceridemia, low HDL-C, or central obesity, as shown in Table 1.

### 3.3. Associations between ApoA5 Level and Metabolic Profiles

Through the Pearson correlation analysis, we found that the serum ApoA5 level was not significantly correlated with the metabolic profiles or liver function, as shown in Table 2. Next, we divided participants into four groups according to the quartiles of the ApoA5 concentration to explore the relationship of the serum ApoA5 level with NAFLD, metabolic profiles, and the prevalence rate of NAFLD and metabolic syndrome in detail. We found that the TG level had a tendency to increase from quartile one (Q1) to quartile three (Q3), while it showed a downward trend in the quartile four (Q4). Likewise, no significant differences were observed either. However, the prevalence rate of hypertriglyceridemia showed an upward trend in individuals with a serum ApoA5 level of Q1 to Q3 and then declined in Q4, showing a significant inverted “U-shaped” trend after adjusting for the confounding factors (*P*=0.043), as shown in Table 3. Notably, individuals with higher serum ApoA5 levels were more likely to suffer from hyperglycemia (*P*=0.046).

## 4. Discussion

NAFLD seriously threatens the human health and is one of the main causes of chronic liver disease worldwide, NAFLD was demonstrated to be closely related to metabolic syndrome, which is characterized by obesity, dyslipidemia, and insulin resistance [8, 21, 24, 25]. But to date, the public understanding about/of NAFLD remains very limited [8]. This status is driving us to conduct a research on this disease. ApoA5, an apolipoprotein discovered in recent years, has been confirmed to play a crucial role in the lipid metabolism, especially in the TG metabolism [21, 26, 27]. A study of the South Korean men reported that, in patients with hyperglycemia or coronary artery disease, serum ApoA5 was positively correlated with TG, while in patients with normal TG, it was negatively correlated [28]. Similarly, a Japanese study showed that, in male patients with type 2 diabetes, ApoA5 was also positively correlated with TG but negatively correlated in healthy controls [29]. While the association of the serum ApoA5 level, metabolic syndrome, and NAFLD in the general population of China is still unclear. The association between the serum ApoA5 level and TG, however, remains uncertain.

In this research, after systematically investigating the association of ApoA5 level, metabolic syndrome, and NAFLD, we found that serum ApoA5 levels have no significant correlation with metabolic syndrome but we observed a higher level of ApoA5 in patients with hyperglycemia, which is contrary to what Ishihara et al. once reported [29]. Moreover, the prevalence of hyperglycemia was increased in the Q1 of the ApoA5 level, suggesting that ApoA5 is closely related to insulin resistance, which may be probably attributed to the potent effect of ApoA5 on TG. In addition, we also found a significantly higher level of ApoA5 in males than in females, whereas the other studies have reported a higher ApoA5 level in females than in males in healthy volunteers [29, 30]. The reasons for these discrepancies remain unclear, and a large sample of research is needed to confirm our findings.

Additionally, our study also indicated that the ApoA5 level has no significant correlation with NAFLD. We suspected that this phenomenon occurs because ApoA5 is mainly released into peripheral circulation with low concentrations. Meanwhile, we also failed to detect the significant correlation between the serum ApoA5 concentration and TG levels or other metabolic characteristics. But interestingly, when the participants were divided into four groups according to the quartile of the ApoA5 level, an inverted “U-shaped” correlation relationship between the ApoA5 level and the prevalence of hypertriglyceridemia was observed, which was partly in line with the previous studies conducted in Korea and Japan [28, 29]. At present, the specific mechanism of this inverted “U-shaped” correlation pattern has not been revealed yet. We speculated that when serum ApoA5 is relatively low, the high TG levels may have stimulated the ApoA5 secretion and be released into circulation (positive correlation). However, when the secretion of ApoA5 reaches a certain threshold, the availability of the serum ApoA5 is higher, which is beneficial to promote the metabolism and reduce the level of TG (negative correlation).

## 5. Conclusion

However, the limitations of our study have to be discussed and documented in the literature. First, this is a cross-sectional observational study; thus, causality cannot be inferred. Second, it is a single-center study with a relatively small sample size. Therefore, it is necessary to increase the sample size in order to get more accurate experimental data to clarify our conclusion.

In spite of the above limitations, we first found that the ApoA5 levels and the prevalence of hypertriglyceridemia are in an inverted “U-shaped” correlation, but there is no significant difference between the ApoA5 levels, NAFLD, and metabolic syndrome.

## Figures and Tables

**Table 1:** The association between the ApoA5 level and gender and the metabolic characteristics.

		ApoA5 (*μ*g/ml)
Gender	Male (*n* = 200)	29.3 ± 4.5
	Female (*n* = 317)	28.5 ± 4.7
	*P*	0.04

Metabolic syndrome	Hyperglycemia	29.4 ± 4.8
	Normal	28.6 ± 4.6
	*P*	0.075

Metabolic syndrome	Hypertension	28.3 ± 5.7
	Normal	28.8 ± 4.6
	*P*	0.32

Metabolic syndrome	Hypertriglyceridemia	28.5 ± 4.5
	Normal	28.7 ± 5.1
	*P*	0.58

Metabolic syndrome	Low HDL-C	28.6 ± 5.0
	Normal	28.9 ± 4.3
	*P*	0.76

*Note*. Significant difference as *P* < 0.05.

**Table 2:** Associations between ApoA5 level and metabolic profiles.

Indexes	ApoA5 level	
	*β*	*P* value
Age (years)	0.039	0.379
Smoking	−0.024	0.683
Hypertension	−0.086	0.108
Diabetes	0.029	0.621
Alanine aminotransferase	0.006	0.895
Aspartic acid	−0.046	0.294
Uric acid	0.084	0.058
Fasting blood glucose	0.077	0.081
Triglyceride	−0.008	0.849
Cholesterol	−0.044	0.321
HDL	−0.037	0.408
LDL	−0.022	0.622

*Note*. *β*: correlation coefficient. Significant difference as *P* < 0.05.

**Table 3:** The quartiles of ApoA5.

Quartile	ApoA5	Hypertension	Diabetes	Alanine aminotransferase	Aspartic acid	Fasting blood glucose	Triglyceride	Cholesterol	HDL	LDL
25	25.54	0.00	0.00	13	17	4.83	0.86	4.05	1.2	2.27
50	28.65	0.00	0.00	17.6	20.7	5.15	1.15	4.63	1.37	2.78
75	31.99	1.00	0.00	26	24.2	5.55	1.67	5.32	1.59	3.39

## Data Availability

Data supporting the findings of this study are available from the corresponding author.
